RETRACTED

# Long non-coding RNA TPTEP1 inhibits hepatocellular carcinoma progression by suppressing STAT3 phosphorylation

**DOI:** 10.1186/s13046-019-1193-0

**Published:** 2019-05-09

**Authors:** Hongda Ding, Junpeng Liu, Ruoyao Zou, Pengrui Cheng, Yang Su

**Affiliations:** Department of the fifth General Surgery, ShengJing Hospital of China Medical University, No. 36 Sanhao road, Shenyang, 110004 China

**Keywords:** Hepatocellular carcinoma, Long non-coding RNA, Cisplatinum, Signal transducer and activator of transcription 3, TPTEP1

## Abstract

**Background:**

Hepatocellular carcinoma (HCC) is still the most common cause of tumor-related death worldwide and accumulating studies report that long non-coding RNAs (LncRNAs) are closely related with HCC development, metastasis and prognosis. Cisplatinum, a well-known chemotherapeutic drug, has been widely used for treatment of numerous human cancers including HCC. This study aimed to investigate the differential expressions of LncRNAs in HCC cells treated with cisplatinum and its underlying mechanism.

**Methods:**

The differential expressions of LncRNAs in HCC cells treated with cisplatinum were determined by RNA-seq. The roles of TPTEP1 in HCC development by applying gene function gain and loss analysis in MHCC97H and QYG-7703 cell lines were detected by quantitative real-time polymerase chain reaction (qRT-PCR), cell proliferation, colony formation, cell invasion and flow cytometry assays. The underlying mechanism of TPTEP1 sensitizing hepatocellular carcinoma cells to cisplatinum was examined by RNA-pull down, western blotting, subcellular fractionation, RNA immunoprecipitation and dual luciferase reporter assays. The effect of TPTEP1 on tumorigenesis in vivo was performed with a subcutaneous xenograft mouse model of HCC. In addition, TPTEP1 expression was detected in clinical tumor tissue samples by qRT-PCR.

**Results:**

LncRNA TPTEP1 was highly expressed in cisplatinum-treated HCC cells, which sensitizes hepatocellular carcinoma cell to cisplatinum-induced apoptosis. TPTEP1 overexpression inhibited, while TPTEP1 knockdown promoted HCC cell proliferation, tumorigenicity and invasion. Furthermore, TPTEP1 exerted its tumor suppressing activities by interacting with signal transducer and activator of transcription 3 (STAT3) to inhibit its phosphorylation, homodimerization, nuclear translocation and down-stream genes transcription. Moreover, TPTEP1 overexpression obviously inhibits tumor masses in vivo in a subcutaneous xenograft mouse model of HCC and TPTEP1 is frequently downregulated in HCC tissues, compared to its corresponding pre-tumor tissues.

**Conclusion:**

LncRNA TPTEP1 inhibits hepatocellular carcinoma cells progression by affecting IL-6/STAT3 signaling. Taken together, our findings suggest a tumor suppressing role of TPTEP1 in HCC progression and provide a novel understanding of TPTEP1 during the chemotherapy for HCC.

RETRACTED

**Electronic supplementary material:**

The online version of this article (10.1186/s13046-019-1193-0) contains supplementary material, which is available to authorized users.

## Background

Hepatocellular carcinoma (HCC) is a highly aggressive malignancy with a poor prognosis [1]. According to the World Health Organization (WHO), HCC is the fifth most common type of cancer with over 700,000 new cases diagnosed every year and the second commonest leading cause of cancer death with an annual death rate of 788,000 people all over the world [2, 3]. Although improvements in HCC treatment, including surgery, radiation therapy, chemotherapy, and immunotherapy, HCC patient still has a poor prognosis with high rates of metastasis and postoperative recurrence, thus the 5 year survival rate is less than 50% [4]. Therefore, better understanding of the underlying molecular mechanism of HCC and developing highly effective treatments for HCC are greatly urgent.

Long non-coding RNAs (LncRNAs) are more than 200 nucleotides long with little or no protein-coding capacity [5]. LncRNAs have been identified to play critical roles in various physiological and pathological processes, including organ development, immunity, organismal viability, tumorigenesis and tumor progression [6–8]. LncRNAs exert their roles by regulating gene transcription in *cis* or *trans*, modulating mRNA processing, post-transcriptional control and protein activity, or organizing nuclear domains [9, 10]. Nowadays, increasing studies have shown that a class of LncRNAs are dysregulated in HCC and closely related with tumorigenesis, metastasis, prognosis or diagnosis [11]. For example, LncRNA HULC accelerates liver cancer by inhibiting PTEN via autophagy cooperation to microRNA15a [12]. LncRNA UFC1 promotes the progression of HCC through interacting with the mRNA stabilizing protein HuR and enhancing β-catenin expression [13]. Our recently study have reported that LncRNA PVT1 inhibits interferon-α mediated therapy for HCC by interacting with signal transducer and activator of transcription 1 (STAT1) [14]. Although lots of LncRNAs have been annotated, most still remain functionally undefined characterized.

Cisplatinum, a well-known chemotherapeutic drug, has been widely used for treatment of numerous human cancers including bladder, head and neck, lung, ovarian, liver, and testicular cancers by interfering with DNA repair mechanisms, causing DNA damage, and subsequently inducing apoptosis in cancer cells [15]. Recently, accumulating evidence indicates that LncRNAs are involved in the process of cisplatinum-induced apoptosis of cancer cells and resistance to chemotherapy by altering the expression of genes at various levels [16]. For example, LncRNA LINC00161 sensitizes osteosarcoma cells to cisplatin-induced apoptosis by regulating the miR-645-IFIT2 axis [17]. LncRNA MEG3 suppresses glioma cell proliferation, migration, and invasion by acting as a competing endogenous RNA of miR-19a [18]. Moreover, LncRNAs are reported to be novel biomarkers for differentiating between cisplatin-resistant and cisplatin-sensitive ovarian cancer [19]. For example, knockdown of LncRNA HOTAIR sensitizes HCC cell to cisplatin by suppressing the STAT3/ABCB1 signaling pathway [20]. Whether other LncRNAs are involved in cisplatinum-induced HCC cell apoptosis and its underlying mechanisms are still unknown.

RETRACTED

In the present study, we investigated the differential expressions of LncRNAs in HCC cells treated with cisplatinum by RNA-seq and identified that LncRNA TPTEP1 was highly expressed in cisplatinum-treated HCC cells. The high level of TPTEP1 sensitizes hepatocellular carcinoma cell to cisplatinum-induced apoptosis. TPTEP1 overexpression inhibited while TPTEP1 knockdown promoted HCC cell proliferation, tumorigenicity and invasion. We revealed that TPTEP1 exerted its tumor suppressing activities by interacting with signal transducer and activator of transcription 3 (STAT3) to inhibit its phosphorylation, homodimerization, nuclear translocation and down-stream gene transcription. Our findings suggest a tumor suppressing role of TPTEP1 in HCC progression and provide a novel understanding of TPTEP1 during the chemotherapy for HCC.

## Methods

### Ethics statement

This study was approved by the Ethics Committee of ShengJing Hospital of China Medical University. All study participants provided written informed consents.

### Collection of specimens

A total of 32 matched samples of primary HCC and adjacent non-cancerous liver tissues (Additional file 1: Table S1) were obtained from ShengJing Hospital of China Medical University. This study was approved by the ethics committee of our hospital, and all participants signed informed consent forms in this study. No patients had received chemotherapy or radiotherapy prior to surgery. HCC and normal tissue specimens were obtained immediately after surgical resection and stored at − 80 °C for further analysis.

### Cells, siRNAs, plasmids and reagents

The human HCC cell lines, including HepG2, SMMC-7721, QGY-7703, Huh-7, MHCC97h, SNU-449 and Sk-hep1, and L02 human normal liver cell line were purchased from American Type Culture Collection (ATCC) or Cell Bank of Shanghai Institute of Biochemistry and Cell Biology, Chinese Academy of Sciences (Shanghai, China), and all cells were cultured in Dulbecco’s Modified Eagle’s Medium (DMEM) supplemented with 10% fetal bovine serum (FBS) and 1% penicillin/streptomycin at 37 °C with 5% CO2 in a humidified incubator. siRNAs against LncRNA LINC01088, AK03516, AC003104.1, LINC00261, RP11–17803.2, SMDA5-AS1, TPTEP1, IDH1-AS1 and LINC00341 were synthetized by GenePharma (Shanghai, China). siRNAs sequences are available in Additional file 1: Table S2. Full-length LncRNA TPTEP1 (NR_001591.1), TPTEP1–2 (1-1080 bp), TPTEP1–3 (534-1483 bp), and TPTEP1–4 (1-500 bp) were amplified by PCR, using primers shown in Additional file 1: Table S2, and then subcloned into pcDNA3.1. STAT3 (full length) (KR710556.1), STAT3 NTD (N-terminal domain), STAT3 NTD + CC + DBD (N-terminal domain+Coiled-coil domain+DNA binding domain), STAT3 △DBD (NTD + CC + LK + SH2 + TA) (N-terminal domain+Coiled-coil domain+DNA binding domain+ Linker domain+Src homology-2 domain+Tail domain), STAT3 DBD + LK + SH2 + TA (DNA binding domain+Linker domain+Src homology-2 domain+Tail domain), STAT3 DBD (DNA binding domain,) constructs were cloned into a pCMV-Flag vector using primers shown in Additional file 1: Table S2. Cisplatinum was purchased from Beyotime (Shanghai, China).

RETRACTED

### RNA-seq and computational analysis

QGY-7703 cells seeded into a 6-well plate were treated with cisplatinum (30μg/ml) for 0, 3, 6 or 12 h. The cells were then collected and lysed in TRIzol reagent (Thermo Fisher Scientific) and total RNAs extraction was conducted according to the manufacturer’s protocol. RNA-seq was performed at the Sequencing and Non-Coding RNA Program at the RiboBio (Guangzhou, China) using Hiseq3000 (Illumina, USA). LifeScope v2.5.1 was used to align the reads to the genome, generate raw counts corresponding to each known gene, and calculate the RPKM (reads per kilobase per million) values.

### Transfection

Cells (5 × 10^5^ cells/well) were cultured in 6-well plates until 60% confluent, and then transfected with plasmids (4 μg/well) or siRNAs (20 nM/well) using Lipofectamine 3000 (Invitrogen) according to the manufacturer’s protocol. Following transfection, cells were incubated in a humidified chamber supplemented with 5% CO_2_ at 37 °C. 24 h after transfection, cells were harvested for RT-qPCR and Western blotting assay.

### Apoptosis assay

Cells seeded into a 6-well plate were transfected with siRNAs. After 24 h, the cells were further treated with 30μg/ml cisplatinum or not for for 24 h, and then cell apoptosis assay was detected using Annexin V-APC/7-AAD apoptosis kit (Lianke, China) by flow cytometry, according to the manufacturer’s instructions. The cells undergoing apoptosis are Annexin V positive.

RETRACTED

### Quantitative real-time PCR (qRT-PCR)

Cells seeded into a 6-well plate were transfected with siRNAs or plasmids. After 24 h, the cells were further treated with 30μg/ml cisplatinum or not for for 24 h, and then harvested. Total RNA was extracted from each sample, using RNA Isolater Total RNA Extraction Reagent (Vazyme, China). For extraction of RNA from the cytoplasm and nucleus, the SurePrep Nuclear or Cytoplasmic RNA Purification Kit (Thermo Fisher Scientific) was used according to the manufacturer’s protocols. RNA from each sample was reverse-transcribed into cDNA using the PrimeScript RT reagent kit (Takara, China). qRT-PCR was performed using the 7500 real-time PCR system (Applied Biosystems), with AceQ qPCR SYBR Green Master Mix (Vazyme, China). The obtained data were normalized to GAPDH expression levels in each sample. The primers for qRT-PCR were listed in Additional file 1: Table S2.

### Construction of stable cell lines

To obtain cell lines stably overexpressing TPTEP1, MHCC97h cells were infected with lentivirus carrying TPTEP1 gene (LV-TPTEP1) or control lentivirus (LV-Control) (Igebiotech, Guangzhou, China). To study the knockdown effects of TPTEP1, QGY-7703 cells were infected with lentivirus carrying shRNA against TPTEP1 (ShRNA-TPTEP1) or control shRNA (ShRNA-Control) (Igebiotech, Guangzhou, China). The efficiency of TPTEP1 overexpression or knockdown was confirmed by qRT-PCR.

### Colony formation assay

For cell colony formation assay, TPTEP1-knockdowned QGY-7703 cells or TPTEP1-overexpressed MHCC97h cells seeded in 6-well plates and cultured for 10 days. The medium was changed every 3 days. The cells were fixed with 4% paraformaldehyde and stained with crystal violet. Finally, the colonies were randomly visualized in five fields under a microscope, and the results were expressed as the average number of colonies in every visual field.

### Matrigel invasion assay

After matrigel (BD Biosciences, Shanghai, China) was added on the transwell chamber and clotted, cells (10^6^ cells per well) were seeded into the top chamber in 200 μL serum-free media. The bottom well was added with 600 μL complete medium. After 24 h, the matrigel and the cells on the top chamber were removed with cotton swab. The cells on the lower surface of the insert were fixed 4% paraformaldehyde, stained with 0.1% crystal violet and counted from five randomly selected fields and averaged. Each experiment was performed in triplicate.

### Cell proliferation assay

Cell proliferation was detected by the MTT assay kit (Beyotime, Shanghai, China). Cells were seeded in 96-well plates at a density of 10^3^ cells/well, and then cultured for 1, 2, 3, 4 or 5 days. Subsequently, 10 μL of MTT solution was added to each well, the plates were incubated for 4 h, and the absorbance was measured at 450 nm.

RETRACTED

### RNA pull-down assay

RNA pull-down assays were performed essentially as previously described [14]. Briefly, biotin-labeled TPTEP1 (Sense) or unrelated fragments (Antisense) were obtained by in vitro transcription and biotin RNA labeling mix (Roche, Switzerland). Then the equal amount of biotin-labeled TPTEP1 or unrelated RNA was added as a control to streptavidin dynabeads. QGY-7703 cells lysates were incubated at room temperature for 15 min to immobilize RNA on the streptavidin dynabeads, then supernatant was removed and beads were washed with wash buffer. Samples were then boiled for 10 min at 100 °C in loading buffer. Finally, the samples were subjected into SDS-PAGE and the gel was then stained with the Fast Silver Stain Kit (Beyotime, Shanghai, China). Proteins specially interacting with Lnc TPTEP1 were identified by reverse-phase liquid chromatography coupled with tandem mass spectrometry (ACQUITYTM UPLC-QTOF).

### RNA-binding protein immunoprecipitation (RIP) assay

RIP assays were performed essentially as previously described [14]. In brief, QGY-7703 or MHCC-97H cells were harvested and lysed (5 mM HEPES [pH 7.4], 85 mM KCl, 0.5% NP40, 1 mM DTT, 5 mM PMSF, supplemented with protease inhibitors cocktail (Roche, Switzerland), RNase inhibitors (Invitrogen, USA) for 8 min on ice. After centrifugation, the supernatant was collected and sonicated and 10% of the lysate serves as ‘input’. The remainder of the lysate was incubated with 40 μl protein G-coupled dynabeads (Life Technologies, USA) for 30 min at 4 °C to decrease the background, followed by washing in lysis buffer and adding protein G-coupled dynabeads with 3 μg anti-STAT3 antibody, anti-flag antibody or IgG control, then rotated overnight at 4 °C. RNA was isolated by TRIzol (Invitrogen, USA), incubated with DNase I (Sigma, USA) and reverse-transcribed into cDNA, and subjected to qRT-PCR detection (primers in Additional file 1: Table S2).

### Dual luciferase reporter assay

TPTEP1 overexpressed MHCC97h cells ((LV-TPTEP1) or TPTEP1 knockdowned QGY-7703 cells (ShRNA-TPTEP1) were seeded in 24-well culture plates and then transfected with pGL3-STAT3 plasmids which containing STAT3 response element and pRL-TK plasmid for 24 h. Luciferase activities were measured with Dual-Luciferase Reporter Assay System (Promega) according to the manufacturer’s instructions. Data are normalized for transfection efficiency by dividing Firefly luciferase activity with that of Renilla luciferase.

RETRACTED

### Subcellular fractionation and Western blotting

Cells seeded into a 6-well plate were treated with 30 ng/ml human IL-6 or not for the indicated time. The cytoplasm and nuclear fraction of cells were extracted using a nuclear and cytoplasmic protein extraction kit (Beyotime, Shanghai, China). Whole cell lysates or the nuclear/cytoplasm fractions were subjected to SDS-PAGE and immunoblotting [14]. Primary antibodies against STAT3 (Abcam, USA), phosphorylated STAT3 (p-STAT3) (Abcam, USA), β-actin (Abcam, USA), GAPDH (a cytoplasm fraction maker, Abcam, USA), Histone H3 (a nuclear fraction maker, Abcam, USA), and flag (Beyotime, China) were used.

### Native PAGE

Native PAGE was performed as described in a previous study [21].

### Tumor formation in nude mice

Eighteen 4-week-old male BALB/c nude mice were divided into 3 groups randomly. Each group was composed of 6 mice that were injected with 2 × 10^6^ MHCC97H cells, control MHCC97H cells (LV-Control) or TPTEP1-overexpressed cells (LV-TPTEP1). Five weeks later, all mice were killed and the weight of each tumor was measured. Tumor tissues were integrally stripped out. All animal studies were approved by the Animal Ethics Committee of China Medical University and experiments were conducted according to the National Institutes of Health Guide for the Care and Use of Laboratory Animals.

### In situ hybridization

Paraffin-embedded sections of xenograft tumors from the nude mice were deparaffinized with xylene and rehydrated with 100, 90, 70 and 50% ethanol (5 min each) at room temperature. The samples were digested with proteinase K and fixed in 4% paraformaldehyde for 10 min at room temperature, followed by hybridization with the TPTEP1 probe (RiboBio, Guangzhou, China) at 55 °C overnight and subsequent incubation with HRP-conjugated secondary antibody for 30 min at 4 °C. Diaminobenzidine was used to develop the stain with a colorimetric reaction for 30 min at room temperature, and then the sections was observed under light microscope.

### Immunohistochemistry

Paraffin-embedded sections of xenograft tumors from the nude mice were dewaxed with 100, 90, 70, and 50% alcohol solutions (5 min each at 37 °C), followed by heat-induced repair in 0.01 mol/l citrate buffer (pH 6.0), 20 min of endogenous peroxidase inhibition with 0.3% hydrogen peroxide, 30 min of incubation at room temperature in 20% normal goat serum and overnight incubation at 4 °C with anti-pSTAT3 antibody. The sections were then incubated for an additional 1 h at 37 °C, washed with 0.01 mol/l PBS and incubated for 20 min at 37 °C with HRP-conjugated secondary antibody. After development with 3,3′-diaminobenzidine reagent for 5 min at room temperature, sections were observed for staining under a light microscope. Finally, hematoxylin was used for 30 s of counterstaining; sections were then rinsed with running water for 5 min, hyalinized and mounted with neutral resin prior to observation under light microscope.

RETRACTED

### In vivo metastatic model

Mice were randomly divided into 2 groups (*n* = 6 per group). 5 × 10^5^ control MHCC97H cells (LV-Control) or TPTEP1-overexpressed cells (LV-TPTEP1) were suspended in 0.1 ml PBS and intravenously injected via lateral tail veins of the mice. The mice were sacrificed 4 weeks later, and the fluorescent protein–positive (GFP) metastatic foci in livers and lungs were analyzed by stereoscopic fluorescence microscope (Leica M205FA, Image Source: Leica DFC500, Wetzlar, Germany).

### Statistical analysis

Data were statistically analyzed and graphed using GraphPad Prism 5 (GraphPad Software, San Diego, CA, USA). All results were presented as mean values ± standard deviations. Statistically significant differences between groups were determined by the Student’s t-test. *P < 0.05.

## Results

### Long non-coding RNA TPTEP1 sensitizes cisplatinum-induced apoptosis in HCC cells

Cisplatinum, a well-known chemotherapeutic drug, is widely used for treatment of HCC [15]. Accumulating evidence indicates that LncRNAs are involved in the process of cisplatinum-induced apoptosis of cancer cells and are novel biomarkers for differentiating between cisplatin-resistant and cisplatin-sensitive cancers [16, 19]. In the present study, we analyzed the LncRNA differential expressions in cisplatinum-treated hepatocellular carcinoma QGY7703 cells by RNA-seq (Fig. 1a). 476 LncRNAs are upregulated and 53 LncRNAs are downregulated in cisplatinum-treated QGY-7703 cells after 12 h stimulation, compared to those in cisplatinum-untreated cells (data not shown). Furthermore, we focused on the nine LncRNAs (LINC01088, AK03516, AC003104.1, LINC00261, RP11–17803.2, SMDA5-AS1, TPTEP1, IDH1-AS1 and LINC00341), which were most highly upregulated in HCC cells after 6 or 12 h cisplatinum treatment. To validate the results, these nine LncRNAs were detected by RT-PCR and the results showed that these nine LncRNAs were indeed highly upregulated in cisplatinum-treated QGY-7703 cells (Fig. 1b).

**Fig. 1:** Long non-coding RNA TPTEP1 sensitizes cisplatinum-induced apoptosis in HCC cells. **a** The heatmap was drawn to show the differentially expressed LncRNAs in hepatocellular carcinoma QGY-7703 cells-treated with cisplatinum (30μg/ml) for the indicated time points by RNA sequencing. **b** Relative expression levels of the ten indicated LncRNAs in cisplatinum-treated QGY-7703 cells were analyzed by qRT-PCR. **c** QGY-7703 cells were transfected with the indicated siRNAs for 24 h and then treated with cisplatinum (30μg/ml) for 24 h. The cell apoptotic rates were analyzed by flow cytometry. **d** The relative expression levels of TPTEP1 in the cytoplasm and nucleus of QGY-7703 cells treated with cisplatinum (30μg/ml) or not for 12 h were analyzed by qRT-PCR (TfIIb as the cytoplasmic maker, and NEAT1 as the nuclear maker). **e** The relative expression levels of TPTEP1 in the indicated HCC cell lines and L02 human normal liver cells were analyzed by qRT-PCR. TPTEP1 expression in L02 cells was used for the control. Data are represented as means ± SD (*n* = 3; ^*^represents *P* < 0.05)

To further investigate the effects of these nine upregulated LncRNAs on cisplatinum-induced apoptosis in HCC cells, these LncRNAs were knockdown by specific small interfering RNAs (siRNAs), respectively (Additional file 1: Figure S1A). Flow cytometry analysis showed that LncRNA AK03516 or SMDA5-AS1 knockdown significantly increased cisplatinum-induced apoptosis in HCC cells, while LncRNA RP11–17803.2, TPTEP1, IDH1-AS1 or LINC00341 knockdown notably inhibited, compared to control (Fig. 1c). Among these LncRNAs, TPTEP1 knockdown has the most obviously inhibitory effects on cisplatinum-induced apoptosis. Thus, we mainly focused on the LncRNA TPTEP1 in the following studies.

RETRACTED

The transmembrane phosphatase with tensin homology (TPTE) gene is located on human chromosome 21 and has many homologous copies/pseudogenes on chromosome 13, 15, 21, 22, and Y [22]. TPTEP1 is also called psiTPTE2 located on chromosome 22 and is silenced by DNA methylation in cancers [23]. Our results showed that TPTEP1 is mainly distributed in the cytoplasm, with a small portion in the nucleus (Fig. 1d). Besides, cisplatinum treatment evidently increased TPTEP1 expression in both cytoplasm and nucleus. Moreover, TPTEP1 was expressed in HCC cell lines to varying degrees, with the highest level in QGY-7703 cells and the lowest level in MHCC97H cells, compared to L02 human normal liver cell (Fig. 1e). Taken together, our results showed that cisplatinum treatment significantly increases LncRNA TPTEP1 expression in HCC cells, which sensitizes cisplatinum-induced apoptosis.

### Long non-coding RNA TPTEP1 suppresses HCC cell proliferation and invasion

To further investigate the effects of TPTEP1 on HCC cell proliferation, tumorigenicity and invasion, TPTEP1 overexpression (LV-TPTEP1) and knockdown (ShRNA-TPTEP1) cell lines were established by lentiviral infection in QGY-7703 or MHCC97H cells. TPTEP1 upregulation and downregulation were confirmed by RT-PCR (Additional file 1: Figure S1C and D). TPTEP1 overexpression significantly inhibited HCC cell proliferation and colony formation, while TPTEP1 knockdown notably increased (Fig. 2a and b, and Additional file 1: Figure S2A). Furthermore, transwell assays showed that TPTEP1 overexpression significantly inhibited HCC cell invasion, while TPTEP1 knockdown notably enhanced HCC cell invasion (Fig. 2c and Additional file 1: Figure S2B). Moreover, TPTEP1 overexpression or knockdown did not affect HCC cell apoptosis (Fig. 2d), suggesting that the inhibition of HCC cell proliferation and invasion by TPTEP1 was not due to the induction of cell apoptosis. Overall, function gain and loss experiments in hepatocellular carcinoma cell lines indicated that TPTEP1 overexpression inhibited HCC cell proliferation and invasion, whereas TPTEP1 knockdown accelerated HCC cell proliferation and invasion.

RETRACTED

**Fig. 2:** Long non-coding RNA TPTEP1 suppresses HCC cell proliferation and invasion. **a** Cell proliferation was examined by MTT assays in TPTEP1-knockdowned QGY-7703 cells (shRNA- TPTEP1) or TPTEP1-overexpressed MHCC97H cells (LV-TPTEP1) at the indicated time points. The shRNA-Control QGY-7703 cells or LV-Control MHCC97H cells were as control. **b** Tumor colony numbers were examined by colony formation assays in TPTEP1-knockdowned QGY-7703 cells (shRNA-TPTEP1) or TPTEP1-overexpressed MHCC97H cells (LV-TPTEP1). **c** Cell invasive ability was examined by transwell invasion assays in TPTEP1-knockdowned QGY-7703 cells (shRNA-TPTEP1) or TPTEP1-overexpressed MHCC97H cells (LV-TPTEP1). **d** Cell apoptotic rates were analyzed by flow cytometry in TPTEP1-knockdowned QGY-7703 cells (shRNA-TPTEP1) or TPTEP1-overexpressed MHCC97H cells (LV-TPTEP1). Data are represented as means ± SD (*n* = 3; ^*^represents *P* < 0.05)

### Long non-coding RNA TPTEP1 directly interacts with STAT3 to suppress HCC cell progression

To further explore the mechanism underlying TPTEP1 suppresses HCC cell proliferation and invasion, biotin-labeled RNA pulldown accompanied by mass spectrometric assays were performed to investigate the TPTEP1-interacting proteins in HCC cells. Among the potential interacting proteins, a specific protein band at approximately 90 kDa in TPTEP1 pull-down samples was observed and then identified as STAT3 protein by mass spectrometry (Fig. 3a). Numerous studies have reported that interleukin-6 (IL-6)/janus kinase (JAK)/STAT3 pathway is aberrantly hyperactivated in many types of cancer, and such hyperactivation is generally associated with a poor clinical prognosis. In the tumor microenvironment, IL-6/JAK/STAT3 signaling acts to drive the proliferation, survival, invasiveness, and metastasis of tumor cells [24–26]. Thus, we pay attention to STAT3 in the following studies. Subsequently, the interaction between TPTEP1 and STAT3 was confirmed by RIP assays (Fig. 3b). To verify whether TPTEP1 suppresses HCC progression is related to its interacting with STAT3, HCC cells were transfected with pCMV-STAT3 plasmid and then treated with cisplatinum to induce apoptosis. As shown in Fig. 3c, cisplatinum treatment notably triggered HCC cell apoptosis and TPTEP1 overexpression further enhanced cisplatinum-induced apoptosis. Whereas, ectopic expression of STAT3 partly reversed TPTEP1 overexpression-induced cell apoptosis under cisplatinum treatment (Fig. 3c). Consistently, STAT3 overexpression in HCC cells also partly attenuated TPTEP1 overexpression-induced inhibition of cell proliferation and invasion (Fig. 3d and e). Taken together, these results demonstrated that LncRNA TPTEP1 directly interacts with STAT3 to suppress HCC cell progression.

RETRACTED

**Fig. 3:** Long non-coding RNA TPTEP1 directly interacts with STAT3 to suppress HCC cell progression. **a** Biotin labeled TPTEP1 was generated through in vitro transcription, and incubated with QGY-7703 lysate for RNA pulldown, and the denoted band of TPTEP1 (Sense) was identified as STAT3 by Mass spectrum. **b** The interactions between TPTEP1 and STAT3 were detected by RIP assays in QGY-7703 and MHCC97H cells. **c** Cell apoptotic rates were analyzed by flow cytometry in TPTEP1-overexpressed QGY-7703 cells (LV-TPTEP1) with or without STAT3 overexpression (pCMV-STAT3) under cisplatinum treatment. **d** Cell prolifiration was examined by MTT assays in TPTEP1-overexpressed QGY-7703 cells (LV-TPTEP1) with or without STAT3 overexpression (pCMV-STAT3) **e** Cell invasive ability was examined by transwell invasion assays in TPTEP1-overexpressed QGY-7703 cells (LV-TPTEP1) with or without STAT3 overexpression (pCMV-STAT3). Data are represented as means ± SD (*n* = 3; ^*^represents *P* < 0.05)

### Domain analysis of interaction between STAT3 and TPTEP1

To further identify the functional domain within TPTEP1 responsible for interacting with STAT3, we cloned a series of deletion constructs of TPTEP1, and then performed RNA pull-down assays. The results showed that the left arm (1 to 500 bp) of TPTEP1 was responsible for the interaction with STAT3 (http://rna.tbi.univie.ac.at/; Fig. 4a). Besides, we also cloned a series of Flag-tagged STAT3 deletion constructs to identify its TPTEP1-binding domain by RIP assay. The results showed that the DNA binding domain (DBD) of STAT3 was responsible for the interaction with TPTEP1 (Fig. 4b).

**Fig. 4:** Domain analysis of interaction between STAT3 and TPTEP1. **a** The STAT3-binding domain in TPTEP1 was identified by RNA pulldown assays in QGY-7703 cells. Left, the structure of TPTEP1 (http://rna.tbi.univie.ac.at/). Right above, the in vitro transcribed full-length TPTEP1 and deleted fragments showing the correct sizes. Right below, immunoblotting analysis of STAT3 in protein samples pulled down by the different TPTEP1 constructs. **b** The TPTEP1-binding domain in STAT3 was identified by RIP assays in QGY-7703 cells. Left, immunoblotting analysis of full-length STAT3 and the domain-truncated fragments. Middle, diagrams of full-length STAT3 and the domain-truncated fragments. Right, QGY-7703 cells were transfected with the indicated STAT3-truncated vectors for 24 h ang then the interactions between TPTEP1 and STAT3 truncated fragments were detected by RIP assays. Data are represented as means ± SD (*n* = 3; ^*^represents *P* < 0.05)

RETRACTED

### Long non-coding RNA TPTEP1 inhibits STAT3 transcriptional activity

To investigate the biological significance of the interaction between TPTEP1 and STAT3, the STAT3 transcriptional activity was detected by luciferase reporter assays in TPTEP1 overexpressed or knockdown HCC cells. The results showed TPTEP1 overexpression significantly depressed the luciferase activity of STAT3 response element, whereas TPTEP1 knockdown notably increased (Fig. 5a). Furthermore, TPTEP1 overexpression evidently inhibited the mRNA and protein expression of MCL1, cyclin D1, Bcl-xl and IL-6, which are the downstream factors in the IL-6/ JAK/STAT3 signaling pathway [27], while TPTEP1 knockdown enhanced these genes mRNA and protein expression (Fig. 5b). Moreover, the TPTEP1 fragments containing the STAT3-interacting ability showed evident inhibitory effects on the proliferation and invasion of HCC cells (Fig. 5c and d). Overall, these results demonstrated that TPTEP1 inhibits STAT3 transcriptional activity in HCC cells.

**Fig. 5:** Long non-coding RNA TPTEP1 inhibits STAT3 transcriptional activity. **a** The luciferase activity of STAT3 response element was detected by Luciferase assays in TPTEP1-knockdowned or TPTEP1-overexpressed QGY-7703 cells. **b** The mRNA (left panel) and protein (right panel) expression levels of MCL1, cyclinD1, Bcl-xl and IL6 were detected by qRT-PCR assays or western blotting in TPTEP1-knockdowned or TPTEP1-overexpressed QGY-7703 cells. **c** and **d** Cell proliferation **c** and invasive ability **d** were detected by MTT assays or transwell invasion assays in QGY-7703 cells infected with the lentivirus expressing full-length TPTEP1, the deletion fragments, or the control. Data are represented as means ± SD (*n* = 3; ^*^represents *P* < 0.05)

### Long non-coding RNA TPTEP1 inhibits STAT3 phosphorylation, homodimerization and nuclear translocation is partly dependent on IL-6

STAT3 transcriptional activity depends on its phosphorylation, homodimerization and nuclear translocation [27]. Thus, we further investigated whether TPTEP1 affected STAT3 phosphorylation, homodimerization and nuclear translocation in HCC cells. Western blotting analysis showed that IL-6 stimulation significantly induced STAT3 phosphorylation in the control HCC cells, and TPTEP1 knockdown furthermore augmented IL-6-induced STAT3 phosphorylation in HCC cells (Fig. 6a), and also strengthened cisplatinum-induced STAT3 phosphorylation in HCC cells (Additional file 1: Fig. S3A). Besides, as expected, TPTEP1 overexpression evidently suppressed IL-6-induced STAT3 phosphorylation in HCC cells (Fig. 6a). Furthermore, TPTEP1 knockdown significantly enhanced IL-6-induced phosphorylated STAT3 nuclear translocation in HCC cells, while TPTEP1 overexpression evidently inhibited (Fig. 6b and Additional file 1: Figure S3B). Since TPTEP1 suppresses the transcription of IL-6 (Fig. 5b) which is well known to induce STAT3 phosphorylation [27], we further explored whether TPTEP1 inhibits STAT3 phosphorylation is dependent on IL-6 or not. We then examined the TPTEP1 expression under IL-6 stimulation and found that IL-6 stimulation did not obviously affect TPTEP1 expression (Additional file 1: Figure S4A). Moreover, through transfection with specific shRNA-against IL-6, we found that both knockdown of TPTEP1 and IL-6 could partly attenuate TPTEP1 knockdown-induced STAT3 phosphorylation (Additional file 1: Figure S4B), suggesting that TPTEP1 inhibits STAT3 phosphorylation is partly dependent on IL-6.

RETRACTED

**Fig. 6:** Long non-coding RNA TPTEP1 inhibits STAT3 phosphorylation, homodimerization and nuclear translocation. **a** TPTEP1-knockdowned QGY-7703 cells or TPTEP1-overexpressed MHCC97H cells were stimulated with IL-6 (30 ng/ml) for the indicated times. The protein expression levels of STAT3 and phosphorylated STAT3 (p-STAT3) were detected by Western blotting (β-actin as loading control). **b** TPTEP1-knockdowned QGY-7703 cells or TPTEP1-overexpressed MHCC97H cells were stimulated with IL-6 for 6 h. The protein expression levels of STAT3 and p-STAT3 in the cytoplasmic and nuclear fractions were detected by Western blotting (GAPDH as the cytoplasmic maker, and Histone H3 as the nuclear maker). **c** QGY-7703 cells were stimulated with IL-6 for 24 h and then the relative expression levels of TPTEP1 interacted with STAT3 were detected by RIP assays. **d** TPTEP1-knockdowned QGY-7703 cells (Left) or TPTEP1-overexpressed MHCC97H cells (Right) were stimulated with IL-6 for 6 h and then the mono and dimer forms of p-STAT3 protein expressions were detected by Native PAGE and Western blotting. Data are represented as means ± SD (*n* = 3; ^*^represents *P* < 0.05)

In addition, RIP analysis showed that IL-6 stimulation significantly augmented the interaction between STAT3 and TPTEP1 (Fig. 6c), and TPTEP1 knockdown or overexpression evidently enhanced or suppressed phosphorylated STAT3 homodimerization (Fig. 6d). Overall, these results indicated that TPTEP1 inhibits STAT3 phosphorylation, homodimerization and nuclear translocation in HCC cells is partly dependent on IL-6.

RETRACTED

### Long non-coding RNA TPTEP1 inhibits tumor masses in mouse and is frequently downregulated in HCC tissues

To explore the effect of TPTEP1 on tumorigenesis in vivo, we generated a xenograft model by subcutaneously implanting MHCC97H cells in nude mice. Nude mice were randomly divided into 3 groups with 6 mice in each group (blank group, LV-Control and LV-TPTEP1) and injected, respectively, with MHCC97H cells, control lentivirus-infected MHCC97H cells, and TPTEP1 overexpressed MHCC97H cells. No obviously differences between the body weights of mice were observed in the three groups (Additional file 1: Figure S5), and TPTEP1 overexpression caused less tumor formation and significantly decreased tumor size compared with blank group or LV-Control group (Fig. 7a and b). Besides, in situ hybridization and immunochemistry analysis showed that phosphorylated STAT3 (p-STAT3) was highly expressed in the tumor tissues of blank group or LV-Control group, while TPTEP1 overexpression evidently suppressed p-STAT3 expression in the tumor tissues (Fig. 7a). Moreover, in vivo metastatic assays showed that TPTEP1 overexpression decreased the number of metastatic liver and lung nodules (Fig. 7c). In addition, we further examined the TPTEP1 expression in 32 pairs of HCC and their corresponding non-tumorous liver tissues by qPCR and found that TPTEP1 was frequently downregulated in the HCC tissues as compared with the non-tumorous tissues (Fig. 7d). Besides, TPTEP1 was apparently decreased in 71.8% of the HCC samples (Fig. 7e). Overall, these results indicate that TPTEP1 inhibits tumor masses in mouse and is frequently downregulated in HCC tissues.

**Fig. 7:** Long non-coding RNA TPTEP1 inhibits tumor masses in mouse and is frequently downregulated in HCC tissues. **a** TPTEP1 overexpression significantly inhibits tumor masses in vivo in a subcutaneous xenograft mouse model of HCC. Left, representative images of xenograft tumors from the nude mice. Middle, expression analysis of p-STAT3 in tumor tissues of each group by immunochemistry (× 200 magnification). Right, expression analysis of TPTEP1 in tumor tissues of each group by in situ hybridization (× 200 magnification). **b** Comparison of tumor weights from each group of nude mice. **c** Number of liver and lung metastatic foci in each group. **d** The copy numbers of TPTEP1 were determined in 32 pairs of HCC tissues and adjacent normal tissues using qRT-PCR. **e** Fold change of TPTEP1 copy number variations in 32 paired tissues. Data are represented as means ± SD (^*^represents *P* < 0.05)

RETRACTED

## Discussion

LncRNAs have been found to participate in hepatocellular carcinoma development by affecting multiply aspects of biological activities in HCC cells. Through interacting with PRMT5 (arginine methyltransferase 5) and blocking ubiquitin/proteasome dependent degradation to enhance its protein stability, LINCO1138 acts as an oncogenic driver in HCC [28]. LncRNA PVT1, which is up-regulated in HCC tissues, promotes stem cell-like property and proliferation of HCC cells by enhancing an RNA-binding protein NOP2 stability [29]. By activating NOTCH2 signaling, LncAKHE cooperated with YEATS4 to promote HCC progression [30]. These studies all focus on the microarray analysis of HCC tissues to find the differential expressed LncRNAs.

In the present study, we screened the differential expressed LncRNAs in cisplastinum-stimulated HCC cells and for the first time found LncRNA-TPTEP1 participates in cisplastinum-induced HCC cell apoptosis by suppressing STAT3 phosphorylation. Moreover, through performing cell proliferation, invasion and apoptosis analysis, we found TPTEP1 could inhibit HCC cell proliferation and invasion but have no effect on HCC cell apoptosis. It seems contradictory to previous results that TPTEP1 partly mediates cisplastinum-induced HCC cells apoptosis [23]. This contradiction maybe attribute to the basal expression of TPTEP1 in HCC cells is low and the difference of TPTEP1 mature form with or without cisplatinum treatment. TPTEP1 has been reported to have 3 transcript variants and be silenced by DNA methylation in cancers of the kidney, liver, lung, and stomach [23]. Besides, TPTEP1 expression could be recovered by DNA demethylation and/or histone deacetylase inhibition [23]. Nowadays, many studies show that chemotherapy could alter DNA Methylation in cancers [31] and DNA methylation of genes are involved in cisplatinum sensitivity in cancer cells [32, 33]. Whether TPTEP1 enhances cisplastinum-induced HCC cell apoptosis is associated with alteration of TPTEP1 DNA methylation and whether any transcript variants of TPTEP1 are affected in HCC cells with cisplastinum stimulation need further investigation in the following studies.

Activated classical IL-6/STAT3 signaling is commonly related to HCC developed from liver injury and inflammation [34] and induces OCT4/NANOG expression to confer poor prognosis of HBV-related hepatocellular carcinoma [35]. Tumor-associated macrophages promotes human hepatocellular carcinoma stem cells expansion by activating IL-6/STAT3 signaling [36]. Above studies indicate the important role of IL-6/STAT3 signaling in HCC progression. In our study, through performing RNA pull down and subsequent mass spectrometric analysis, we found TPTEP1 directly binds to STAT3 and suppresses IL-6-induced STAT3 phosphorylation. Combined with RIPs and transcriptional analysis, we also demonstrated that TPTEP1 suppresses STAT3 nuclear translocation and STAT3 transcriptional activity. Since IL-6 is well known to induce STAT3 phosphorylation and then phosphorylated STAT3 translocated into nucleus to promote IL-6 transcription [27], it is suggested that TPTEP1 specifically interacts with STAT3 to inhibit STAT3 transcriptional activity, resulting in reducing IL-6 expression, which further blocks STAT3 phosphorylation. Indeed, our results demonstrated that TPTEP1 inhibiting STAT3 phosphorylation is partly dependent on IL-6. However, the detailed mechanism of TPTEP1 suppressing STAT3 phosphorylation has not been explored. Whether STAT3 phosphorylation promoting elements were inhibited or STAT3 phosphorylation inhibitory factors were activated by TPTEP1 is still unknown. Besides, whether TPTEP1 interacting with STAT3 destroys the interaction between STAT3 and other related kinase is also needed to be investigated in the future studies.

RETRACTED

## Conclusions

Our study firstly identified that TPTEP1 sensitizes hepatocellular carcinoma cells to cisplatinum by interacting with STAT3 to inhibit IL-6 induced STAT3 phosphorylation. Although the underlying mechanisms still need to be elucidated in further studies, our findings suggest a tumor suppressing role of TPTEP1 in HCC progression and provide a novel understanding of TPTEP1 during the chemotherapy for HCC.

## Additional file

Additional file 1: **Figure S1.** (A) Knockdown efficiencies of siRNAs against the ten indicated LncRNAs in QGY-7703 cells were detected by qRT-PCR. (B) Ratio of RPKM (reads per kilobase per million mapped reads) value from ribosomal profiling of each indicated gene in QGY-7703.(C and D) Relative RNA levels of TPTEP1 in QGY-7703 cells infected with the lentivirus expressing shRNA against TPTEP1 (shRNA-TPTEP1) (C), or in MHCC97H cells infected with the lentivirus expressing TPTEP1 (LV-TPTEP1) were detected by qRT-PCR (n=3; *represents *P* < 0.05). **Figure S2.** Cell proliferation (A) and invasive ability (B) were examined in shRNA-Control QGY-7703 cells and TPTEP1-knockdowned QGY-7703 cells (shRNA-TPTEP1-2, another TPTEP1 shRNA used to avoid off-target effects) (n=3; *represents *P* < 0.05). **Figure S3.** (A) STAT3 and p-STAT3 protein expressions in QGY-7703 cells infected with lenti-shRNA-TPTEP1 and then treated with cisplatinum (CS) were detected by Western blotting. (B) STAT3 and p-STAT3 protein expressions in the cytoplasmic and nuclear fractions in QGY-7703 cells infected with lenti-shRNA-TPTEP1 and then stimulated with IL-6 were detected by Western blotting (GAPDH as the cytoplasmic maker, and Histone H3 as the nuclear maker). **Figure 4.** (A) TPTEP1 expressions in IL-6 stimulated QGY-7703 cells were detected by qRTPCR. (B) STAT3 and p-STAT3 protein expressions in TPTEP1-knockdowned QGY-7703 cells transfected with shRNA-IL6 and then stimulated with IL-6 for 6 h were detected by Western blotting (n=3; *represents *P* < 0.05). Figure S5. BALB/c nude mice were divided into 3 groups randomly, and were injected with MHCC97H cells (NC), control MHCC97H cells (LV-Control) or TPTEP1-overexpressed cells (LV-TPTEP1). Five weeks later, the body weights of mice were monitored (n=6; *represents *P* < 0.05). **Table S1.** Clinicopathological Characteristics of the human samples used in this study. **Table S2.** Primers used in this study. (DOCX 321 kb)

RETRACTED

## Abbreviations

HCC: Hepatocellular carcinoma
IL-6: interleukin-6
JAK: janus kinase
LncRNAs: long non-coding RNAs
qRT-PCR: quantitative real-time polymerase chain reaction
STAT3: signal transducer and activator of transcription 3
TPTE: transmembrane phosphatase with tensin homology
